The article "Correlation of Glucose and Lipid Metabolism Levels and Serum Uric Acid Levels with Diabetic Retinopathy in Type 2 Diabetic Mellitus Patients" was published in 2022. Journal: Emerg Med Int.

# Correlation of Glucose and Lipid Metabolism Levels and Serum Uric Acid Levels with Diabetic Retinopathy in Type 2 Diabetic Mellitus Patients

**DOI:** 10.1155/2022/9201566

**Published:** 2022-07-21

**Authors:** Tiantian Li, Yan Wu

**Affiliations:** Department of General Practice, The First People's Hospital of Lianyungang, Lianyungang 222000, Jiangsu, China

## Abstract

**Objective:**

The aim of this study was to observe the association between the development of diabetic retinopathy (DR) in type 2 diabetes mellitus (T2DM) and the levels of glucose and lipid metabolism and serum uric acid (SUA) levels.

**Methods:**

A retrospective analysis was performed on 97 patients with T2DM who were admitted to our endocrinology department from June 2019 to April 2021 with complete data; the patients were divided into DR and no DR groups (NDR) according to the presence or absence of DR. Their clinical history and biochemical test indexes were collected, and the fundus was examined by fundus photography and the fundoscopic examination method, and the vascular diameter was measured by using a computer software. All clinical data, medical history, and biochemical test indexes were compared between the two groups, and logistic regression was used to analyze the risk factors of DR.

**Results:**

The duration of DM disease, fasting blood glucose (FBG), glycosylated hemoglobin, type A1C (HbA1c) levels, cholesterol (TC), triacylglycerol (TG), low-density lipoprotein cholesterol (LDL-C), and SUA levels were higher in the DR group than those in the NDR group, and the differences were significant (*P* < 0.05). The difference between the NDR group and the DR group in terms of gender, age, BMI, DBP, SBP, family history of DM, FINS, and HDL-C levels was not significant (*P* > 0.05). The results of multifactorial analysis showed that the four variables of DM duration, HbA1c, TG, and SUA were still risk factors for the development of DR (*P* < 0.05). Further receiver operating characteristic (ROC) analysis showed that the areas under the curves (AUCs) for the duration of DM disease, HbA1c, TG, and SUA to predict the occurrence of DR were 0.740 (95% CI 0.639–0.841), 0.767 (95% 0.672–0.862), 0.721 (95% CI 0.617–0.826), and 0.693 (95% CI 0.588∼0.797), respectively.

**Conclusion:**

The lesions of DR in T2DM patients have a close relationship with the course of DM, HbA1c, TG, and SUA, and the course of DM, HbA1c, TG, and SUA has a good predictive value for the occurrence of DR.

## 1. Introduction

Diabetes mellitus (DM) is a common clinical metabolic disease characterized by chronic and persistent elevation of blood glucose, which can cause damage to multiple tissues and organs, including the heart, eyes, kidneys, nerves, and blood vessels [1, 2]. In recent years, the incidence of diabetes has been increasing in China, and now, it has become the country with the largest number of people with diabetes in the world. It is well known that the danger of diabetes is mainly in its complications, and diabetic retinopathy (DR) is one of the most common diabetic microvascular complications and the leading cause of visual impairment and irreversible blinding disease in the working population [3, 4]. The development of DR is associated with a variety of risk factors as well as biomarkers. According to the literature [5], the severity of DR is associated with the prolonged duration of DM, elevated glycated hemoglobin levels, proteinuria production, hyperglycemia, glucose levels, and dyslipidemia. However, it has been clinically found that even though the above factors have been strictly controlled, they do not completely stop the progression of DR, and there may be other factors involved in the pathogenesis of DR. Therefore, it is important to identify new risk factors that may affect DR and thus slow down its progression.

The article "Correlation of Glucose and Lipid Metabolism Levels and Serum Uric Acid Levels with Diabetic Retinopathy in Type 2 Diabetic Mellitus Patients" was published in 2022. Journal: Emerg Med Int.

At this stage, the main indicators commonly used in clinical practice to detect the degree of glycemic control and the degree of abnormal glucose metabolism are glycated hemoglobin (HbA1c) and fasting blood glucose (FPG), and the application of these two indicators plays an important role in the treatment of diabetes and in the prevention and treatment of complications [6]. Uric acid is the end product of purine metabolism, and with increasing research on uric acid, it has been found to be biologically active, causing endothelial dysfunction, inflammation, vasoconstriction, and having both positive and negative antioxidant and pro-oxidant stress effects [7]. Serum uric acid (SUA) has been reported to be an independent risk factor for cardiovascular disease and is closely associated with various metabolic syndrome components such as obesity, hyperglycemia, dyslipidemia, and insulin resistance [8, 9]. Studies have shown that SUA is closely related to the development of diabetic nephropathy and uric acid-lowering therapy can reduce proteinuria in patients with type 2 diabetes. There are fewer studies on uric acid and diabetic retinopathy, and the relationship between uric acid and diabetic retinopathy is unclear. Elevated blood lipids can increase glomerular pressure and change vascular resistance, causing abnormalities in the body's metabolism, which is an important indicator of the development of diabetes [10]. In this study, we analyzed the risk factors affecting the occurrence of DR in diabetic patients by testing the glucolipid metabolism level and the blood uric acid level, aiming to provide relevant testing indicators for the prevention of DR in clinical practice.

The article "Correlation of Glucose and Lipid Metabolism Levels and Serum Uric Acid Levels with Diabetic Retinopathy in Type 2 Diabetic Mellitus Patients" was published in 2022. Journal: Emerg Med Int.

## 2. Materials

### 2.1. Study Subject Selection

In this study, clinical data were collected from 97 patients with type 2 diabetes mellitus who were hospitalized between June 2019 and April 2021 in the endocrinology department of our hospital. According to the 2017 American Academy of Ophthalmology Diabetic Retina Guidelines [11], the patients were divided into the DR group (42 cases) and the no DR group (NDR group, 55 cases) according to whether they had DR or not.

### 2.2. Screening Criteria

① No previous primary kidney disease, renal insufficiency, viral hepatitis, leukemia, malignancy, and other diseases that can cause elevated blood uric acid. ② No previous retinal vascular obstruction, atherosclerotic, hypertensive, hematologic or diabetic fundoplication, no retinal detachment, retinal tumor, or other related diseases. ③ No previous medication to promote uric acid excretion or to inhibit uric acid synthesis. ④ Patients who have not been previously treated with kidney dialysis or kidney transplantation. ⑤ Patients with no febrile symptoms and no concomitant heart failure, malignancy, or pregnancy on physical examination and ancillary tests. ⑥ With the patient's consent and the ability to perform fundus photography, the resulting images showed clear fundus vascular contours without blurred borders or obscuration.

### 2.3. Diagnostic Criteria for T2DM

The diagnosis of diabetes mellitus was performed according to the 1999 WHO diagnostic criteria [12], i.e., the patient had clinical manifestations of diabetes mellitus. Hyperglycemia: fasting blood glucose (FBG) ≥7.0 mmol/L at any time or plasma glucose ≥11.1 mmol/L or glucose tolerance test (OGTT test) 2-hour glucose ≥11.1 mmol/L.

### 2.4. Research Methodology

#### 2.4.1. General Data Collection

Patients' names, gender, age, hospitalization number, duration of DM, family history of DM, height, weight, and blood pressure (BP) were collected from the medical record management system of our hospital. Patients' height and weight were measured by the same height-weight measuring device in the department, and BMI (weight/height^2^, kg/m^2^) was calculated based on the measured data. BP was measured on the day of admission, after sufficient rest, by the nurses in our department using an electronic blood pressure meter.

#### 2.4.2. Clinical Biochemical Index Collection

All patients fasted from food and water for more than 8 hours, and venous blood was drawn early the next morning. Serum glucolipid metabolic indexes were measured using an automatic biochemical analyzer, including FBG, HbA1c, cholesterol (TC), triacylglycerol (TG), low-density lipoprotein cholesterol (LDL-C), and high-density lipoprotein cholesterol (HDL-C) levels, and fasting insulin (FINS) level was measured by radioimmunoassay. SUA levels were measured by the uricase peroxidase ascorbate oxidase method.

The article "Correlation of Glucose and Lipid Metabolism Levels and Serum Uric Acid Levels with Diabetic Retinopathy in Type 2 Diabetic Mellitus Patients" was published in 2022. Journal: Emerg Med Int.

#### 2.4.3. Fundus Radiographs

Diabetic retinopathy was examined by our ophthalmologists using optical coherence tomography (OCT) and fundus fluorescence angiography (FFA) to diagnose the presence or absence of DR, and patients were grouped according to the diagnosis.

### 2.5. Statistical Analysis of the Experiment

Statistical analysis of the data of this experiment was performed using SPSS17.0 software. The results of normally distributed measures were expressed as mean ± standard deviation, i.e., $\bar{x}\pm s$, and the *t*-test was used for comparison between the groups. The statistical data were expressed as the number of cases (percentage, %), and the *χ*^2^ test was used to compare between the groups. The risk factors for RD were analyzed by logistic regression analysis. For statistical analysis, differences were considered statistically significant at *P* < 0.05.

## 3. Results

### 3.1. Comparison of General Information between the Two Groups

Finally, 42 patients diagnosed with DR were included in the DR group, and the remaining 55 patients were included in the NDR group. We collected basic information on admission such as name, gender, age, hospitalization number, duration of DM, family history of DM, height, weight, and blood pressure (BP) of all patients and compared some of them. The results showed that the duration of DM was significantly higher in the DR group than that in the NDR group (*P* < 0.05). The comparison between the NDR and DR groups in terms of gender, age, BMI, DBP, SBP, and family history of DM is shown in Table 1. The differences were not significant (*P* > 0.05).

### 3.2. Comparison of Glucose Metabolism Levels between the Two Groups

We examined the serum glucose metabolism levels of all patients and the indexes including FBG, HbA1c, and FINS and analyzed the differences between the NDR and DR groups, and the results showed that the FBG and HbA1c levels in the DR group were significantly higher than those in the NDR group (*P* < 0.05). The FINS levels in the NDR and DR groups were not significantly different (*P* > 0.05) (Figure 1).

### 3.3. Comparison of Lipid Metabolism Levels and Blood Uric Acid Levels between the Two Groups

We examined the serum lipid metabolism and SUA levels of all patients. Lipid metabolism includes TC, TG, LDL- C, and HDL-C. The differences between the NDR and DR groups were analyzed, and the results showed that TC, TG, LDL-C, and SUA levels were significantly higher in the DR group than those in the NDR group (*P* < 0.05). HDL-C levels in the NDR and DR groups were not significantly different (*P* > 0.05) (Figure 2).

The article "Correlation of Glucose and Lipid Metabolism Levels and Serum Uric Acid Levels with Diabetic Retinopathy in Type 2 Diabetic Mellitus Patients" was published in 2022. Journal: Emerg Med Int.

### 3.4. Multiple Regression Analysis of DR Risk Factors

In this study, logistic multiple regression was used to analyze the magnitude of the effect of each factor on DR. The abovementioned study showed that the duration of DM, FBG, HbAlc, TC, TG, LDL-C, and SUA may all be related to the occurrence of DR. Logistic multiple regression analysis was performed to adjust for risk factors, with the occurrence of DR as the dependent variable, and the duration of DM, FBG, HbAlc, TC, TG, LDL-C, and SUA as independent variables. The results showed that the four variables of DM duration, HbA1c, TG, and SUA were still risk factors for the occurrence of DR (*P* < 0.05), with OR values of 1.110 (95% CI 1.020–1.207, *P* < 0.001), 2.721 (95% CI 1.181–6.271, *P*=0.014), 1.033 (95% CI 1.018∼1.047, *P*=0.008), and 3.013 (95% CI 1.277∼7.110, *P*=0.004), respectively, as shown in Tables 2 and 3.

### 3.5. ROC Analysis of DR Risk Factors

According to the results of multifactor regression analysis, the duration of DM, HbA1c, TG, and SUA were risk factors for DR. To further investigate whether the duration of DM disease, HbA1c, TG, and SUA could be used as predictors of DR, we did ROC analysis of DR with the occurrence of DR as the dependent variable and the durations of DM disease, HbA1c, TG and SUA as separate independent variables. The results showed that the AUCs of the duration of DM, HbA1c, TG, and SUA to predict the occurrence of DR were 0.740 (95% CI 0.639–0.841, *P* < 0.001), 0.767 (95% 0.672–0.862), 0.721 (95% CI 0.617 to 0.826, *P* < 0.001), and 0.693 (95% CI 0.588 to 0.797, *P*=0.001), respectively (Table 4, Figure 3).

## 4. Discussion

DR is one of the microvascular complications of diabetes mellitus, with a high clinical prevalence, and is the main cause of vision loss in middle-aged and elderly people. The high incidence and high disability rate of DR not only have a serious impact on the physical and mental health of patients, but also greatly increase the economic expenses of families and impose a heavy burden on the healthcare system and society [13]. It has been suggested [14] that the site of chronic complications in diabetes is associated with the activation of pathways such as long-term hyperglycemia, hyperlipidemia, abnormal glucose metabolism, and oxidative stress due to abnormal lipid metabolism. It is now generally accepted in studies that the risk of developing DR in patients with DM increases linearly when the duration of the disease exceeds 10 years and that the duration of DM is an independent risk factor for the development of DR [15]. The results of this study are consistent with previous literature reporting a book. In this study, the mean duration of DM in the DR group was 13 years, which was significantly higher than that in the NDR group, while multiple factors suggest that the duration of DM is a risk factor for the development of DR. This reminds us that when the duration of DM is more than 10 years, we should be alert to the occurrence of DR, and we can improve the prognosis of patients by providing health education, developing an early screening program for related complications, and timely detection and treatment.

The article "Correlation of Glucose and Lipid Metabolism Levels and Serum Uric Acid Levels with Diabetic Retinopathy in Type 2 Diabetic Mellitus Patients" was published in 2022. Journal: Emerg Med Int.

Hyperglycemia is an important factor in triggering DR. A large number of studies [16–18] have confirmed that long-term chronic hyperglycemia is the main cause of chronic complications, and HbA1c is a sensitive indicator reflecting glycemic control, and some literature has reported that glycemic control in diabetic patients is closely related to the occurrence and development of DR. In this study, the HbA1c levels of DR patients were significantly higher than those of MD-NDR patients, and the results of multifactorial analysis and correlation analysis confirmed that HbA1c was the main risk factor for the development of DR in MD patients, which was more consistent with the results of previous studies. A chronic hyperglycemic environment can lead to nonenzymatic glycosylation of proteins in the body, resulting in thickening of the basement membrane and even causing vascular occlusion impeding oxygen diffusion, causing retinal hypoxia, and thus leading to the development or exacerbation of DR. This shows that HbA1c plays an important role in the pathogenesis of DR [19, 20].

Patients with MD are often associated with disorders of lipid metabolism, and elevated lipids will promote the extent of DR and the development of diabetic macular degeneration, which is mainly manifested by macular hard exudates in the early clinical stage [21–23]. The results of this study showed that there were statistically significant differences in blood TC, TG, and LDL-C levels in DR patients compared with those in the NDR group, and multifactorial analysis showed that TG was a risk factor for the development of DR and had a good predictive value for the development of DR. Elevated lipids cause tissue peroxidation through the nonenzymatic glycosylated polyol pathway, leading to damage to the vascular wall and endothelial dysfunction, causing hemodynamic changes, retinal tissue hypoxia, and consequent microcirculatory disorders, leading to a series of microvascular lesions such as atherosclerosis and hemorrhage in the fundus, and eventually the formation of microthrombi, which destroy the retinal barrier and cause the development of retinopathy [24].

The article "Correlation of Glucose and Lipid Metabolism Levels and Serum Uric Acid Levels with Diabetic Retinopathy in Type 2 Diabetic Mellitus Patients" was published in 2022. Journal: Emerg Med Int.

As research has progressed, a large number of investigators have concluded that SUA levels are associated with increased risk in patients with DR. A prospective study [25] found that glucose and uric acid concentrations were significantly higher in the vitreous humor of MD patients compared to controls, while patients with progressive DR had higher levels of uric acid in the vitreous humor compared to those with nonprogressive DR This suggests that uric acid levels in diabetic patients may be associated with the development and progression of DR, as seen in a growing number of studies suggesting a correlation between SUA and DR. The results of this study showed that the level of SUA was significantly higher in the DR group than in the NDR group, and the results of multifactorial analysis showed that SUA was an independent risk factor for the development of DR in patients with DM. We further performed ROC analysis on the risk of DR occurrence and showed that the AUC of SUA to predict DR was 0.693 (95% CI 0.588–0.797, *P*=0.001), indicating that SUA has some risk predictive value for the occurrence of DR. Most studies [26, 27] suggest that UA may be involved in the development of DR through several aspects such as pro-oxidative stress, proneoangiogenesis, reduced protective effects of promelanocytes, proinsulin resistance, and promotion of retinal atherosclerosis, but the mechanisms involved have not been fully elucidated due to their complexity and variety.

In this study, a retrospective analysis of 97 T2DM patients revealed that the lesions of DR in T2DM patients had a close relationship with the duration of DM, HbA1c, TG, and SUA. Therefore, in clinical work, we should pay attention to the disease course, glucose and lipid metabolism level, and SUA level of DM patients, strengthen patient health education, improve 'patients' lifestyle, actively control 'patients' blood glucose and blood lipid levels, and if necessary, give UA-lowering drug treatment, in order to comprehensively improve the metabolic disorders of DM patients and to prevent or delay the development of DM-related chronic complications.

## Figures and Tables

**Figure 1:** Comparison of glucose metabolism levels between the two groups (*n*$\bar{x}\pm s$). (a∼c) FBG (mmol/L), HbA1c (%), and FINS (mIU/L), respectively; ^∗^ indicates a significant difference between the DR and NDR groups (*P* < 0.05).

**Figure 2:** Comparison of lipid metabolism levels and blood uric acid levels between the two groups (*n*$\bar{x}\pm s$). (a∼e) HDL-C (mmol/L), TC (mmol/L), TG (mmol/L), LDL-C (mmol/L), and SUA (*μ*mol/L), respectively; ^∗^ indicates significant differences between the DR and NDR groups (*P* < 0.05).

The article "Correlation of Glucose and Lipid Metabolism Levels and Serum Uric Acid Levels with Diabetic Retinopathy in Type 2 Diabetic Mellitus Patients" was published in 2022. Journal: Emerg Med Int.

**Figure 3:** ROC analysis of DR risk factors. (a∼c) The predictive value of DM disease duration, HbA1c, TG, and SUA on the occurrence of DR, respectively.

**Table 1:** Comparison of general information between the two groups ($\bar{x}\pm s$; (*n*, %)).

Information		NDR group (*n* = 55)	DR group (*n* = 42)	*t*/*χ*^*2*^ value	*P* value
Sex (M/F)		31/24	27/15	0.622	0.430
Age (years)		56.24 ± 10.13	58.60 ± 9.00	1.192	0.236
Course of DM (years)		9.25 ± 2.99	12.24 ± 4.07	4.172	0.0001
BMI (kg)		25.42 ± 4.26	26.22 ± 3.13	1.024	0.309
DBP (mmHg)		83.20 ± 12.24	80.48 ± 14.06	1.017	0.312
SBP (mmHg)		136.29 ± 20.24	139.50 ± 21.51	0.753	0.453

Family history of DM	Yes	30 (54.55)	24 (57.14)	0.065	0.799
	No	25 (45.45)	18 (42.86)		

**Table 2:** Multifactor assignment method.

Influencing factors	Assignment
Course of DM	Continuous variables
FBG	Continuous variables
HbA1c	Continuous variables
TC	Continuous variables
TG	Continuous variables
LDL- C	Continuous variables
SUA	Continuous variables

**Table 3:** Multiple regression analysis of DR risk factors.

Indicators	*B*	SE	Wald *x*^2^	*P* value	OR	95% CI
Course of DM	0.104	0.043	32.236	<0.001	1.110	1.020∼1.207
FBG	0.534	0.381	2.170	0.139	1.706	0.808∼3.600
HbA1c	1.001	0.426	6.724	0.014	2.721	1.181∼6.271
TC	1.120	1.105	0.523	0.471	3.065	0.351∼26.730
TG	0.032	0.007	10.138	0.008	1.033	1.018∼1.047
LDL-C	0.423	0.326	0.826	0.343	1.527	0.806∼2.892
SUA	1.103	0.438	15.235	0.004	3.013	1.277∼7.110

**Table 4:** ROC analysis of DR risk factors.

Indicators	AUC	95% CI	*P* value	Cutoff	Sensitivity (%)	Specificity (%)
Course of DM	0.740	0.639∼0.841	<0.001	0.353	57.10	78.20
HbA1c	0.767	0.672∼0.862	<0.001	0.437	61.90	81.80
TG	0.721	0.617∼0.826	<0.001	0.409	50.00	90.90
SUA	0.693	0.588∼0.797	0.001	0.337	81.00	53.70

## Data Availability

The data in this study will be made available from the authors upon reasonable request.
